# Efficient Framework for Detection of COVID-19 Omicron and Delta Variants Based on Two Intelligent Phases of CNN Models

**DOI:** 10.1155/2022/4838009

**Published:** 2022-04-21

**Authors:** Mustafa Ghaderzadeh, Mohammad Amir Eshraghi, Farkhondeh Asadi, Azamossadat Hosseini, Ramezan Jafari, Davood Bashash, Hassan Abolghasemi

**Affiliations:** ^1^Student Research Committee, Department and Faculty of Health Information Technology and Management School of Allied Medical Sciences, Shahid Beheshti University of Medical Sciences, Tehran, Iran; ^2^School of Electrical Engineering, Iran University of Science and Technology, Tehran, Iran; ^3^Department of Health Information Technology and Management, School of Allied Medical Sciences, Shahid Beheshti University of Medical Sciences, Tehran, Iran; ^4^Department of Radiology, Baqiyatallah University of Medical Sciences, Tehran, Iran; ^5^Department of Hematology and Blood Banking, School of Allied Medical Sciences, Shahid Beheshti University of Medical Sciences, Tehran, Iran; ^6^Pediatric Congenital Hematologic Disorders Research Center, Shahid Beheshti University of Medical Sciences, Tehran, Iran

## Abstract

**Introduction:**

While the COVID-19 pandemic was waning in most parts of the world, a new wave of COVID-19 Omicron and Delta variants in Central Asia and the Middle East caused a devastating crisis and collapse of health-care systems. As the diagnostic methods for this COVID-19 variant became more complex, health-care centers faced a dramatic increase in patients. Thus, the need for less expensive and faster diagnostic methods led researchers and specialists to work on improving diagnostic testing.

**Method:**

Inspired by the COVID-19 diagnosis methods, the latest and most efficient deep learning algorithms in the field of extracting X-ray and CT scan image features were used to identify COVID-19 in the early stages of the disease.

**Results:**

We presented a general framework consisting of two models which are developed by convolutional neural network (CNN) using the concept of transfer learning and parameter optimization. The proposed phase of the framework was evaluated on the test dataset and yielded remarkable results and achieved a detection sensitivity, specificity, and accuracy of 0.99, 0.986, and 0.988, for the first phase and 0.997, 0.9976, and 0.997 for the second phase, respectively. In all cases, the whole framework was able to successfully classify COVID-19 and non-COVID-19 cases from CT scans and X-ray images.

**Conclusion:**

Since the proposed framework was based on two deep learning models that used two radiology modalities, it was able to significantly assist radiologists in detecting COVID-19 in the early stages. The use of models with this feature can be considered as a powerful and reliable tool, compared to the previous models used in the past pandemics.

## 1. Introduction

Two years after the emergence of coronavirus, while many countries were experiencing an overall decline in cases, COVID-19 variants have led to a spike in deaths and hospitalizations in some other countries. Since late November 2021, a new wave of uncertainty and panic of the pandemic has spread around the world, as the number of cases of coronavirus 2019 (COVID-19) has increased dramatically, especially in the southern part of Africa, Europe, and East of Asia. A new type of SARS-CoV-2, B.1.1.529, was identified by the World Health Organization as a type of concern and named Omicron [1]. The Omicron and Delta variants of COVID-19 were one of the most dangerous versions of the virus whose prevalence in Europa and then west of Asia led to a record surge in incidence and mortality rates. According to the CDC, the Omicron and Delta variants spread twice as easily as the Alpha variants and are several times more contagious than the previous variants; thus, in January 2022, the Omicron variant becomes the dominant variant worldwide. If not diagnosed in time, it can affect the entire lung in less than a few days, after which patients may suffer from hypoxia due to pulmonary fibrosis that can lead to death [1–8]. Thus, the first and most important step in controlling the COVID-19 latest variants is rapid diagnosis and monitoring of disease cases. Although PCR is the gold standard for diagnosing COVID-19, the long turnaround time for PCR results caused disease high progression and worsening in the case of the Omicron and Delta variants. On the other hand, people with the disease can infect many people until the result is announced as a source of disease transmission. Moreover, research on Omicron and Delta variants has shown that the PCR test has a high rate of false negatives; this is one of the main problems of this diagnostic test that reduces its sensitivity and has irreparable consequences for patients. Radiological tests, including CT and X-ray tests, are one of the most important tools for monitoring suspect COVID-19 cases (7). CT scans are more sensitive and specific than chest radiographs, and in many cases, lung fibrosis was seen on CT even before the onset of clinical symptoms and positive PCR test [4, 7–9]. However, due to the high cost of CT scan, as well as the radiation of this radiological method, the protocol for diagnosing begins with examining the X-ray condition of the suspected COVID-19 case, and then, effects of GGO in the lungs are referred to CT scan centers for a more accurate diagnosis and quantification of the extent of lung involvement. Notably, as the number of patients at radiology diagnostic centers increased, researchers began to use artificial intelligence to design tools to assist clinicians and radiologists in the diagnosis of COVID-19 [9–11].

Since the beginning of the pandemic, numerous studies have used machine learning and in-depth research to design models for the diagnosis and classification of different COVID-19 variants. Of note, many of these states of the art have been very successful. However, all of these studies used a single radiology modality to diagnose and classify COVID-19, and studies have shown that diagnosis based on a radiographic image has some flaws; for instance, it differs significantly from individual diagnosis and also has a high probability of error in detecting COVID-19 from other abnormalities. In the present study to cover this defect, based on diagnostic protocols, we presented a two-phase model to distinguish cases of COVID-19 from other cases such as pneumonia and healthy cases.

## 2. Methods

In the present study, by reviewing previous research using deep learning and the success of convolution neural networks in extracting the features of different images of chest radiographs in COVID-19, designation and implementation of two network developed pretrained CNNs for accurate detection of smart framework patients is suggested.

### 2.1. Dataset

The dataset used for this study included two categories of data classes: CT scan and X-ray images. In this research, an X-ray database has been obtained from the Kaggle [12, 13] to train the initial phase of the framework, and also, a limited local database has been used to test this phase. In addition, a comprehensive database including CT scan images for training and testing of the model's second phase has been collected from the radiology centers of Tehran University Hospitals, so that it is completely native. The definitive status of this dataset cases has been determined after the PCR test.  Table 1 shows the dataset used in this research.

### 2.2. Proposed Method

In order to identify patients with COVID-19 in the early stages of the disease, a comprehensive framework based on two CNNs has been presented. The present framework contains two developed models which are placed in a row as two phases for accurate diagnosis of the COVID-19 Omicron and Delta variants.

#### 2.2.1. Data Preparation

Research has shown that the extraction of hidden patterns in medical images using machine algorithms is not solely due to CNN models, but much of this achievement comes from the use of appropriate image preprocessing techniques (24). In the first stage of the research, i.e., the data preparation stage, the dataset images were received in DICOM format as the output of the PAC system from the diagnostic center, as well as the Kaggle website. However, the characteristics of the images were different since the images were collected from different local diagnostic centers with dissimilar radiology equipment. To address this issue, first, it is converted to a single gray channel space (grayscale), and then, each image is repeated three times to be prepared as dummy RGB channels. Finally, X-ray images in sizes 224, 224, and 3 and CT scan images in sizes 255, 255, and 3 were resized for standard model input.

#### 2.2.2. Data Normalization

One of the most important steps of preprocessing is data normalization, which plays a vital role not only in image convergence speed but also in increasing training speed. For this purpose, first, the global average and the standard deviation of the pixel surface for all images were calculated, and then, the data were normalized using Equation (1), where *x* is the global average of the set of images *X*, *σ* is the standard deviation, and *ε* = 1*e* − 10  is a small value to prevent the denominator from becoming zero.

(1) $$\begin{array}{c} X_{i}=\frac{X_{i}-\bar{x}}{\sigma +\varepsilon }. \end{array}$$

After normalization, with the aim of standardizing the images to achieve a single uniform scale for the input of the deep neural network model, the pixel values of each image were first scaled by transferring to the interval [0,255] and then by converting to the interval [0,1].

#### 2.2.3. Data Augmentation

Since CNN networks are data-driven, as the amount of data increases, the efficiency of these processing units improves due to the maximum coverage of the feature space [14, 15]. At this stage, data were added to the train dataset category using the methods of vertical flip, horizontal flip, and rotation range = 30. This augmentation was done in such a way that those images that are most similar to the original images of the dataset are obtained, and images that are not like noise for the model are produced. Also, the images should not significantly differ from the characteristics of the original images while retaining the defining characteristics of the disease. X-ray and CT-augmented images were produced and were added for both phases of the model.

Before feeding the data to the networks, all the images of the dataset were shuffled so that the network does not necessarily see the data of a particular class during each iteration, and in fact, each category contains images with different tags from both classes of COVID-19 and non-COVID-19 cases including different pneumonias. The datasets in this study were categorized according to Table 2 to be used for training and testing for models.

#### 2.2.4. Transfer Learning

Deep learning models are inherently data-driven. But because the size of the dataset in real-world problems is much smaller than the standard dataset used in deep learning, the concept of transitional learning as a way to overcome data scarcity limit can be used to reinforce the class process. Transfer learning is the transfer of knowledge from one domain to another using weight trained in the previous domain. Traditionally on CNN, the primary multilayer weight matrices are frozen in training the second issue, and only the remaining layers are fined. This process works well when both problems in the overlap area have low-level properties. It is impossible to build a model from scratch due to computational constraints or time constraints, so to implement the concept of transfer learning, pretrained models are tools that help artificial intelligence engineers develop a deep neural network based on an existing framework [16–18] In the present study, since the two datasets ImageNet and COVID-19 belong to nonoverlapping domains, the weights trained from the ImageNet dataset for initialization of the model matrix weights of this study were used. Compared to the random weighting of the layers, this method allows for a better initial weighting of the layers.

#### 2.2.5. Feature Extraction

Feature extraction is one of the key actions in the performance of classification algorithms. In the field of disease diagnosis, this action should be done with more sensitivity in order to correctly extract and display the characteristics that determine the anomalies. In this study, after examining the image features extraction methods, it was found that a special pretrained network was able to extract the features more optimally for each type of research dataset.

*(1) DenseNet201*. DenseNet201 utilizes a dense network that provides models with easy and highly efficient parametric training due to the possibility of reusing features by different layers that increase diversity at the next layer input and improve performance [19]. The DenseNet201 has shown remarkable performance on varying datasets such as ImageNet and CIFAR-100. To improve the connectivity in the DenseNet201 model, direct connections from all preceding layers to all subsequent layers are introduced.

*(2) ResNet152*. ResNet networks have been proposed as a family of multiple deep neural networks with similar structures but different depths. ResNet introduces a structure called a residual learning unit to reduce the destruction of deep neural networks. The structure of this unit is a feed network with a shortcut connection that adds new inputs to the network and generates new outputs. The main advantage of this unit is that it helps to achieve better classification accuracy without increasing the complexity of the model [20].

## 3. Results and Discussion

### 3.1. Proposed Model

A two-phase framework that is inspired by the COVID-19 diagnostic guideline and the diagnostic process in hospitals was designed and implemented. In order to achieve a framework with maximum accuracy and minimum error, two pretrained models were selected for feature extraction from both kind of radiology images. In the proposed method, after reviewing and evaluating most common pretrained networks, including VGG-19, Xception, InceptionV3, ResNet50V2, VGG-16, InceptionResNetV2, and DenseNet201, it was determined that DenseNet-201, a successful torsion architecture in the field of medical image feature engineering, has the best performance in extracting X-ray image features. Therefore, the feature extraction block based on this architecture was selected for the first phase of the proposed model. This architecture has fewer learnable parameters than *most common architectures*; therefore, it has less time complexity than other models. In the second phase, the ResNet152 pretrained network with a high-efficiency was used for CT image feature extraction.  Figure 1 describes the proposed framework in detail. The details of the feature extraction block and transition layers are exactly the same as the original references. In both phases of the proposed framework, the classifier layers used the optimal combination of layers to classify the properties. The topology of these layers was a dense layer, then batch normalization, a dropout layer to avoid overfitting, and the final layer which included an activation function called ReLU (rectified linear unit).

The output of the first phase of this framework, as a screening tool based on X-ray images, can report COVID-19 cases with high accuracy. But if X-ray cannot identify the infectious patient or the output of the first phase is suspicious and contradicts the patient's physical symptoms, according to the physician's opinion, the patient goes through CT scan for a much more accurate diagnosis. CT images taken from the patient are then analyzed using a developed model based on ResNet152 to classify the COVID-19 cases based on the hidden and complex features, and then, these features are classified. At the end of this phase, the output of the images was classified using a classification block developed solely for this phase.  Figure 1 shows a general schematic of the framework. The implementation (source code) of the proposed method is made publicly available at https://github.com/MAmirEshraghi/Deep_Covid19_Detection_Overall_framework.

The feature extraction block is frozen at the beginning of the training phase and starts working inspired by model transfer learning. It first initialized with the weights obtained from the learning on the ImageNet dataset. After training the classification block, the feature extraction block is reactivated and the network fits on the same data again with more repetitions and periods. In this way, while transferring the knowledge gained from the training to the dataset, ImageNet fine-tuned the feature extractor for the specific purpose. In the learning phase, the initial learning rate of 0.0001 and the binary interaction entropy cost function were used. After training the dense layers, the feature extraction block was reactivated, and the network was fitted to the same data again.  Table 3 shows the model parameters of each phase.

### 3.2. Metrics

In the present study, traditional measures to evaluate the performance of the proposed model were used, which are calculated based on a confusion matrix. According to the confusion matrix, specificity and sensitivity to measure and analyze the performance of each proposed model, and overall framework can be calculated. Specificity is the ability of the classifier to correctly identify those without the disease or normal (true negative rate), while sensitivity is the classifier's ability to classify all those with the disease correctly (true positive) [21]. The formulas of the evaluation criteria are given in

(2) $$\begin{array}{c} \text{Sensitivity}=\text{Recall}=\frac{\text{True Positive}}{\text{True Positive}+\text{False Negative}}, \end{array}$$

(3) $$\begin{array}{c} \text{Specificity}=\frac{\text{True Negative}}{\text{True Negative}+\text{False Posetive}}, \end{array}$$

(4) $$\begin{array}{c} \text{Accuracy}=\frac{\text{True Negative}+\text{True Posetive }}{\text{Total Cases}}. \end{array}$$

The confusion matrix is used as one of the performance evaluation indicators in AI models.  Figure 2 depicts the confusion matrix of the model evaluation on the test data and provides a better view of the results on the X-ray test data. The low error rate in this model indicates the high accuracy of the first phase of the model in diagnosing and classifying cases of COVID-19. Analysis of the confusion matrix determined the performance of the first phase of the model was based on public test data and according to Table 4.

The learning curve of the first phase of proposed model for training and validation of datasets is shown in Figure 3. In evaluating the behavior of the proposed model in the management of new validation data, we observed that with increasing epochs, the model reaches lower error rate and therefore increased accuracy for unknown data, indicating that this model has a high potential for detecting new COVID-19 cases from an X-ray images. The mean square error in the detection of all COVID-19 and non-COVID-19 cases among the images in the experimental set was 0.0284.

Since we had a low number of X-ray images available due to the lack of storage of these images in local hospitals, the first phase of the model was trained and tested with public data. To evaluate the performance of the proposed first phase of the model in real-life applications and also to present a comparative evaluation, we tested this phase of the model on a locally available X-ray dataset. This model phase was also tested on native data samples, and the model performance is shown in Table 5.

Figure 4 shows the results of the performance evaluation of the proposed model on 16 random X-ray new samples from the native test suite. In this figure, *N* represents the image index, *P* is the category predicted by the model, and GT indicates the objective truth label. The high accuracy of the model resulted in only one wrong classification out of 16 observations.

In the second phase of the proposed framework, both training and testing are performed with completely native data. In this phase, the performance of the model was calculated using CT category test data, but before those three steps were done, data preprocessing, CT scan image feature extracting, and classifying it according to the customized extended classification block, which included a set of different layers and finally maintaining the parameters of the second phase model. The configuration matrix for this phase is represented in Figure 5, which indicated a low model error on the test data.

According to the confusion matrix in Figure 5, the evaluation indicators of the model can be displayed.  Table 6 shows the metrics of these indicators.

In the second phase of the model, the training curve Figure 6 indicates changes in accuracy and cost during training and validation. In this phase of the model, the training and validation chart is associated with an increase in epochs with reduction in error and increasing in accuracy. Eventually, the validation and training charts converge.

Figure 7 displays the proposed model's evaluation results on 16 random samples from the test dataset. This phase of the model has categorized all sixteen images correctly. Here, *N* is the image index, *P* is the class predicted by the model, and GT is the ground-truth label. Due to the model's high precision, there was no unsuccessful sample prediction to examine the model's possible weaknesses.

The performance of each phase alone achieved acceptable results, but when the two phases were embedded in the proposed framework and tested with local data at the hospital center, it was able to identify all COVID-19 including Omicron and Delta variant cases from other cases including pneumonia or healthy.

## 4. Conclusion

The Omicron and Delta COVID-19 variants can affect the entire lung in less than a few days, so there is a necessity to find more accurate and faster methods to diagnose it with the help of clinicians and health-care systems. This might also impose lower costs on these systems. As WHO emphasized on maximizing diagnostic tests to cover all suspected patients, it is recommended to provide more comprehensive and accessible tests with computer technology-based radiology systems. In the early stages of the Omicron and Delta variants, CT scan of the lungs was not able to show the area of lung consolidation in all cases, or in many cases GGO findings were not observed; accordingly, machine learning models needed to use a combination of radiology modalities for early and faster detection of COVID-19.

In previous studies, data classes were categorized solely on the basis of a CT or X-ray slide using machine learning methods; however, in this method, two radiology modalities were used to classify the cases at the beginning of the disease. Notably, following the complete test of the proposed framework in the teaching hospital under the supervision of a radiologist, it completely identified all cases referred to the hospital and achieved 100% efficiency, suggesting that the proposed framework using two states of the art may probably minimize the error in COVID-19 diagnosis.

By comparing the performance indicators of this research with the network with other state-of-the-art approaches, including traditional deep neural networks and pre-trained networks (Table 7), it can be concluded that the proposed framework in the present study has been able to classify all cases of these variants correctly with higher efficiency.

## Figures and Tables

**Figure 1:** The proposed framework for COVID-19 detection based on two phase of CNN models and radiology modalities.

**Figure 2:** Confusion matrix of the first phase of the model on public test data.

**Figure 3:** The training and validation loss and accuracy of the first phase of proposed model during training. Model converged after 20 epochs with training accuracy and loss of 99.66% and 0.011, respectively, and validation accuracy and loss of 99.08% and 0.045.

**Figure 4:** The first phase performance evaluation results on 16 X-ray random samples. *N*, *P*, and GT are image index, model prediction, ground-truth label, respectively. The green caption indicates accurate prediction, while red shows the inaccurate prediction.

**Figure 5:** Confusion matrix of the second phase of the model on public test data.

**Figure 6:** The training and validation loss and accuracy of the second phase of proposed model during training. Model converged after 10 epochs with training accuracy and loss of 99.7% and 0.011, respectively, and validation accuracy and loss of 99.08% and 0.045.

**Figure 7:** The second phase of proposed model's performance evaluation results on 16 random samples, *N*, *P*, and GT are image index, model prediction, and ground-truth label, respectively. The green caption indicates accurate prediction, while red shows the inaccurate prediction.

**Table 1:** Details on the dataset used for training and evaluating the proposed model.

	Status	No. of samples	No. of patients
X-ray	Public	COVID-19: 3616	COVID-19: 130
		Non-COVID-19: 7200	Non-COVID-19: 240
	Local	COVID-19: 111	COVID-19: 111
		Non-COVID-19: 230	Non-COVID-19: 230
CT scan	Local	COVID-19: 12231	COVID-19: 165
		Non-COVID-19: 2251	Non-COVID-19: 28

**Table 2:** The datasets were categorized according to the table to be used for training and testing for models.

Dataset	Train rate	Validation rate	Test rate
X-ray	82%	9%	9%
CT scan	71%	15%	14%

**Table 3:** Parameters of both phases of the model after tuning.

	Optimizer	Learning rate	Initial learning rate	Decay rate	Decay steps	Loss	Epoch	Batch size
Phase 1	Adam	Exponentially decay	0.0001	0.96	40	Sparse categorical cross entropy	40	32
Phase 2	Adam		0.0001			Sparse categorical cross entropy	30	32

**Table 4:** The evaluation criteria based on the confusion matrix using public X-ray.

Metric	Value
Sensitivity	99
Specificity	98.6
Accuracy	99.09
Precision	99.5

**Table 5:** The evaluation criteria based on the confusion matrix using local X-ray data.

Metric	Value
Sensitivity	99
Specificity	98.6
Accuracy	98.83
Precision	99.5

**Table 6:** The evaluation criteria based on the confusion matrix using local CT scan data.

Metric	Value
Sensitivity	99.7
Specificity	99.76
Accuracy	99.7
Precision	99.8

**Table 7:** Performance comparison of different models for classification of COVID-19.

Model	Accuracy	Precision	Recall
xDNN [22]	97.3	99.1	95.5
DenseNet201 [23]	96.2	96.2	96.2
Modified VGG19 [24]	95.0	95.3	94.0
COVID CT-Net [25]	90.7	88.5	85.0
Contrastive learning [26]	90.8	95.7	85.8
Proposed			
First phase (X-ray data used)	98.83	99.5	99
Second phase (CT data used)	99.7	99.8	99.7
The whole framework	All cases can be classified correctly		

## Data Availability

No data were used to support the findings of this study.
